This article has been retracted.

# Evaluation of the Effect of PDCA in Hospital Health Management

**DOI:** 10.1155/2021/6778045

**Published:** 2021-12-20

**Authors:** Huanmin Qiu, Weiwei Du

**Affiliations:** ^1^Party Committee Office, The First Affiliated Hospital of Suchow University, Suzhou 215006, China; ^2^Propaganda Department of Party Committee, Renmin Hospital of Wuhan University, Wuhan 430060, China

## Abstract

PDCA plays a very important role in the hygienic management of hospital operating rooms. Before the PDCA management from February 2018 to February 2019, routine hygiene management in the operating room was adopted; after the PDCA management from February 2018 to February 2019, PDCA cycle management was adopted. 500 surgical patients were randomly selected from both groups. We compare the quality control checklist scores of hand hygiene management, environmental hygiene management, medical waste management, and disinfection and isolation management in the routine group and the PDCA group. We also compared the detection rate of pathogenic bacteria in surgical incisions of the routine group and the PDCA group and the infection rate of various surgical incisions, air samples, surface samples, disinfectants, and sterilization rates of sterile items. The PDCA group's hand hygiene management score, environmental hygiene management score, medical waste management score, and disinfection and isolation management score were higher than those in the conventional group (*P* < 0.05). The detection rate of pathogenic bacteria in the PDCA group, the infection rate of type I, type II, and type III incisions, and the total infection rate of surgical incisions were lower than those in the conventional group, and the difference was statistically significant (*P* < 0.05). The qualified rate of air samples and surface samples in the PDCA group was higher than that in the conventional group (*P* < 0.05), and the difference in the qualified rate of disinfectants and sterile items between the two groups was not statistically significant (*P* > 0.05). The hygiene management of the operating room adopts PDCA sustainable improvement management measures to effectively increase the qualification rate of disinfection and sterilization, reduce the detection rate of pathogenic bacteria and infection rate of surgical incisions, and strengthen the management quality of hand hygiene, environmental hygiene, medical waste, and disinfection and isolation.

## 1. Introduction

Hospital health management is the key to avoid nosocomial infection. Improving the quality of health management is of great significance to improve medical quality and promote patients' early recovery, which is an important part of hospital management [1]. Studies have pointed out that [2] various pathogenic bacteria are important vectors of infection. When the cleaning and disinfection of the hospital environment are not in place, microorganisms are more likely to survive and reproduce in the medical environment for a long time, which has become an important hidden danger of multidrug resistance and nosocomial infection. PDCA cycle is a management mode with timeliness. It was first conceived by Shewhart and later expanded into a quality control cycle by Dr. Deming in the United States, including four cycle links of P (plan), D (do), C (check), and A (act). It has been widely used in management [3, 4]. This study compared the quality of health management before and after the application of PDCA in the operating room of our hospital and also discussed the effect of PDCA in the health management of the operating room of the hospital. It is reported as follows.

The key contributions of this work are as follows:

1. A literature survey of various existing PDCA algorithms is conducted, and their advantages and disadvantages are analyzed.
2. An effective PDCA optimization model for resource allocation is proposed.
3. A cloud computing environment resource allocation algorithm inspired by PDCA is proposed.
4. The performance of the proposed algorithm is analyzed and compared with other classic algorithms.

The rest of this article is organized as follows.  Section 2 discusses related data and methods, including specific quantitative observation indicators and statistical methods. Then, Section 3 observes the results of the experiment and discusses the summary of the paper and future research directions.

## 2. Data and Methods

### 2.1. Clinical Data

The study was divided into two stages. The first stage was before PDCA management from February 2018 to February 2019. The clinical data of 500 surgical patients were randomly selected from this stage as the routine group. The second stage is after PDCA management, from February 2018 to February 2019. The clinical data of 500 surgical patients were randomly selected as the PDCA group.

There were 295 males and 205 females in the routine group, whose age ranged from 21 to 72 years, with an average of (46.11 ± 6.97) years. In the data used in this article, following cases of respective departments were considered: 153 cases of gynecology, 227 cases of surgery, and 120 cases of orthopedics. Incision types are as follows: 148 cases of type I, 263 cases of type II, and 89 cases of type III. In the PDCA group, there were 278 males and 222 females. The age ranged from 23 to 75 years old, with an average of (45.03 ± 7.82) years old. According to the department classification, his clinic has 130 cases of gynecology, 239 cases of surgery, and 131 cases of orthopedics. Incision types were as follows: 161 cases of class I, 255 cases of class II, and 84 cases of class III. There was no significant difference in gender, age, disease, and surgical incision between the two groups (*P* > 0.05).

### 2.2. Management Method

For the routine group, the routine health management of the operating room, including operating room environmental disinfection, sterilization monitoring, incision infection prevention, disinfection and isolation, hand hygiene, sterile article management, etc., was adopted.

For the PDCA group, PDCA cycle management was adopted.

*Planning Stage* (*P*). PDCA quality control team was established, which was headed by the Department Director and head nurse as the team leader and deputy team leader, and also included 6 team members. Improve the operating room health management system, disinfection system, and reporting system with reference to the code for clinical nosocomial infection prevention and control and quality management [5] and the technical code for hospital disinfection [6]. Analyze the current situation of health management in the operating room, formulate various plans and target control scoring tables around the core factors causing nosocomial infection, including quality control scoring tables such as environmental sanitation, surgical waste management, disinfection, and isolation, and regularly organize training to learn relevant knowledge.

*Implementation Stage* (*D*). PDCA quality control team members are responsible for training the management level of medical staff in the operating room, such as environmental hygiene, hand hygiene, disinfection and isolation, medical waste, and so on, and supervising the implementation of various systems. The team leader and deputy team leader shall use the morning meeting time to carry out “one question a day” for junior doctors, nurses, and anesthesiologists in the department for key links and important knowledge points, confirm the implementation of relevant systems, and jointly supplement learning in case of wrong or incomplete answers. The operating room shall be reasonably arranged, and the room temperature shall be adjusted to 22°C∼24°C and the humidity shall be adjusted to 40%∼60%. All kinds of personnel channels and goods flow were scientifically distributed, and also the placement of medical equipment was reasonably arranged. Sterile operating room, general operating room, infected operating room, restricted area, semirestricted area, and nonrestricted area were strictly divided, and red, yellow, and blue eye-catching signs were, respectively, used. All goods are placed in fixed positions to control cross infection. Before and after the operation, wipe and disinfect the surface and ground of various articles with 0.21% effective chlorine. During the operation, the distance between the sterile table and the operating table was strictly controlled, and the sterile operation procedures were also implemented. The concept of sterility was strengthened in the whole process. Postoperative medical wastes shall be placed in medical waste containers or packaging bags for closed disposal according to categories. Sterile articles shall be managed by special personnel. The identification, validity period, and integrity of sterilized articles shall be checked and registered every day. Optimize the operation of disinfection monitoring in the operating room, pay attention to detail management, register the monitoring and supervision results of daily infection management, and ensure the safety of all links of each operation.

*Inspection Stage* (*C*). In order to achieve the purpose of the experiment, the PDCA team members will check the operation area, sterile materials, disinfectant, and other links every day to ensure that the surgical instruments are complete, the sterile materials and disinfectant have not expired, and they are clean and hygiene. All-round supervision and inspection were conducted every month according to the quality control supervision form of hand hygiene management, environmental hygiene management, medical waste management, and disinfection and isolation management, and 100 points to each supervision form were assigned. The supervision was carried out in various forms of theoretical assessment, on-site inspection, random questioning, and sampling monitoring, and the responsibility of the supervision results was assigned to the person and also linked to the performance. Also, regularly invite relevant personnel of hospital health management to participate in the supervision and review, analyze the health management quality of the operating room in combination with the internal and external evaluation results, and solve the existing problems circularly, so as to achieve the quality control goal.

*Disposal Stage* (*A*). the PDCA team summarized the problems and influencing factors of nosocomial infection in the operating room every month. Also, the characteristics of the department with objective analysis together with the team members were summarized. The team identified deficiencies one by one according to the characteristics of the department, formulated solutions, and incorporated the improvement goals and rectification plans into the next PDCA cycle management model, so as to continuously and systematically improve the health management of the operating room.  Figure 1 shows the brief flowchart of PDCA.  Figure 2 shows the specific implementation diagram of PDCA.  Figure 3 shows the implementation effect diagram of PDCA.

### 2.3. Observation Indicators

The comprehensive effect of operating room hygiene management was compared with the scores of quality control supervision form of hand hygiene management, environmental hygiene management, medical waste management, and disinfection and isolation management in the routine group and PDCA group.

Comparison of pathogen detection rate and infection rate of surgical incision between routine group and PDCA group was conducted.

*Qualification of Disinfection and Sterilization*. Both groups randomly took 500 air samples, object surface samples, disinfectants, and sterile articles during the management period to analyze the qualification of disinfection and sterilization.

In this study, the accuracy (Acc), recall (RE), sensitivity (Sen), and run time analysis model were used to classify the test set. The calculation methods of Acc, RE, and Sen are as follows:

(1) $$\begin{array}{c} \mathrm{Acc=}\frac{\mathrm{TP+TN}}{\mathrm{TP+FN}},\\ \mathrm{RE=}\frac{\mathrm{TP}}{\mathrm{TP+FN}},\\ \mathrm{Sen=}\frac{\mathrm{TP}}{\mathrm{TP+FN}}, \end{array}$$

in which TP represents the number of correct classification results; FN represents the number of missed classifications; TN represents the number of misclassifications; and FP represents the number of wrong classification results.

### 2.4. Statistical Methods

SPSS19.0 was used for statistical analysis. The counting data were expressed in case (%), and *χ*^2^ test was used for comparison. Measurement data ($\bar{x}\pm s$) showed that independent sample *t*-test was adopted for comparison, with *P* < 0.05 as the difference, which was statistically significant.

## 3. Results

### 3.1. Comprehensive Effect of Operating Room Health Management

The scores of hand hygiene management, environmental hygiene management, medical waste management, and disinfection and isolation management in the PDCA group were significantly higher than those in the routine group (*P* < 0.05).  Table 1 shows the comparison of management scores before and after PDCA management in the operating room.

### 3.2. Incision Infection Rate

The detection rate of surgical incision pathogens, the infection rate of classes I, II, and III incision, and the total infection rate of surgical incision in PDCA group were lower than those in the routine group (*P* < 0.05).  Table 2 shows the comparison of pathogen detection rate and infection rate of surgical incision before and after PDCA management in the operating room.

### 3.3. Qualification of Disinfection and Sterilization

The qualified rates of air samples and object surface samples in the PDCA group were higher than those in the routine group (*P* < 0.05). There was no significant difference in the qualified rates of disinfectants and sterile articles between the two groups (*P* > 0.05).  Table 3 shows the comparison of disinfection and sterilization qualification before and after PDCA management in the operating room.

Statistical analysis is performed on the basic clinical features of all patients, as shown in Figure 4. Among all patients, 32 patients (66.67%) were older than 50 years old, 29 patients (60.42%) had left overflow, 45 patients (93.75%) had fertility history, 42 patients (87.5%) had lactation history, and only 8 patients (16.67%) had breast disease history. Among all the patients, 26 patients (54.17%) had serous nipple discharge, 12 patients (25%) had bloody nipple discharge, 8 patients (16.67%) had milky white nipple discharge, and 2 patients (4.17%) had clear water-like nipple discharge.

## 4. Discussion

The health management of the operating room not only is related to the operation effect but also directly affects the risk of nosocomial infection. The management mode used in the past is mostly based on experience summary. With the change of medical counting and management mode, there is a certain degree of inadaptability [7, 8]. Improving the quality of health management in operating room is one of the keys to improve medical quality and reduce the risk of infection. PDCA is a new management concept. The whole process is linked and progressive layer by layer, which plays an obvious role in promoting the management level in all aspects [9, 10].

In this study, PDCA was used in the hygiene management of the operating room. The results showed that the average of hand hygiene management, environmental hygiene management, medical waste management, and disinfection and isolation management in the operating room was significantly improved and the qualified rate of air samples and object surface samples was also greatly improved. The detection rate of pathogens and incision infection rate of the surgical incision were reduced from 13.20% and 9.60% to 4.80% and 3.40%. It is suggested that the application of PDCA in the health management of operating room can effectively improve the quality of health management and reduce the risk of incision infection.

PDCA is a scientific management method. In the planning stage, our plan was to analyze the problems existing in the health management of the operating room and formulate improvement measures. In the implementation stage, according to the formulated improvement measures, the medical staff in the operating room shall be trained in environmental hygiene, hand hygiene, disinfection and isolation, medical waste, and other aspects. In the inspection stage, a supervision mechanism to supervise the implementation of improvement measures was established and summarized according to the assessment results. In the treatment stage, the PDCA team jointly summarized the shortcomings or emerging problems after the implementation of the improvement measures and integrated the improvement measures into the next PDCA cycle, so as to make the health management of the operating room in a state of continuous improvement. Compared with conventional management methods, PDCA has the characteristics of top down. PCDA formed an open loop of problems in the management process, improved methods, and improved new problems, which can improve the implementation of management methods and ensure the implementation of improvement measures, so as to promote the improvement of health management quality [11, 12]. In addition, PDCA has a high restrictive effect on the health management of the operating room. Through the four stages of planning, implementation, inspection, and treatment, all links of the health management of the operating room are integrated into the virtuous circle of planning, measures, evaluation, feedback, and rectification, so as to achieve the expected goal. This process can not only strengthen the risk management awareness of high-risk links but also enhance the disinfection and isolation awareness, hand hygiene awareness, and aseptic operation awareness of operating room staff and finally improve the health management quality of operating room [13, 14]. Some experts believed that [15, 16] the advantage of PDCA is that it is not achieved overnight, but a continuous process. The current problems can be solved through one cycle, and new problems can be solved through the next cycle. Neglected problems in the process of operating room health management can be found over a long period of time, with high timeliness. With the progress of medical technology and the upgrading of management system, we can continuously obtain high health management quality. Foreign studies believe that [3, 17] PDCA can greatly improve the standardization of hand hygiene and the qualified rate of disinfection and sterilization in the operating room, which is consistent with the conclusion of this study. Domestic research by Sun shujun [3, 14, 18] showed that the implementation of hand hygiene management based on PDCA can improve the awareness and compliance of hand hygiene knowledge of operating room nurses and is of great value in reducing operating room infection. According to Zhao Ying's research [1, 5, 19], PDCA can effectively reduce the detection rate of *Staphylococcus aureus* and multidrug-resistant *Acinetobacter* on the surface of hospital environmental objects and strengthen the effect of health management.

## 5. Conclusion

In the paper, PDCA sustainable improvement management measures and prevention management concept are adopted in the health management of the operating room, which can effectively improve the qualified rate of disinfection and sterilization, reduce the detection rate and infection rate of surgical incision pathogens, and strengthen the management quality of hand hygiene, environmental hygiene, medical waste, and disinfection and isolation.

## Figures and Tables

**Figure 1:** The brief flowchart of PDCA.

**Figure 2:** The specific implementation diagram of PDCA.

**Figure 3:** The implementation effect diagram of PDCA.

**Figure 4:** Statistical graph of basic clinical features. (a) Statistical graph of patients' age, overflow side, childbearing history, and breastfeeding history. (b) Statistical graph of the history of breast disease and the proportion of overflow features in patients.

**Table 1:** Comparison of management scores before and after PDCA management in operating room (score, $\bar{x}\pm s$).

Group	Cases	Hand hygiene management	Environmental sanitation management	Medical waste management	Disinfection and isolation management
General group	500	94.64 ± 3.42	93.66 ± 3.20	95.76 ± 3.41	92.19 ± 3.73
PDCA group	500	97.85 ± 2.16	96.31 ± 3.61	98.86 ± 1.01	95.26 ± 4.08
*t* value		17.745	12.283	19.491	12.418
*P* value		0.000	0.000	0.000	0.000

**Table 2:** Comparison of pathogen detection rate and infection rate of surgical incision before and after PDCA management in the operating room (cases, %).

Group	Cases	Pathogen detection rate	Incision infection rate			
			Class I incision	Class II incision	Class III incision	Total infection rate
General group	500	66 (13.20)	5.41 (8/148)	9.13 (24/263)	17.98 (16/89)	48 (9.60)
PDCA group	500	24 (4.80)	1.24 (2/161)	3.53 (9/255)	7.14 (6/84)	17 (3.40)
*χ* ^2^ value		21.538	4.268	6.797	4.570	15.812
*P* value		0.000	0.039	0.009	0.033	0.000

**Table 3:** Comparison of disinfection and sterilization qualification before and after PDCA management in the operating room (score, $\bar{x}\pm s$).

Group	Cases	Qualified rate of air sample	Qualified rate of object surface samples	Qualified rate of disinfectant	Qualified rate of sterile articles
General group	500	466 (93.20)	471 (94.20)	488 (97.60)	494 (98.80)
PDCA group	500	486 (97.20)	489 (97.80)	495 (99.00)	498 (99.60)
*χ* ^2^ value		8.754	8.438	2.932	2.016
*P* value		0.003	0.004	0.087	0.156

## Data Availability

The simulation experiment data used to support the findings of this study are available from the corresponding author upon request.
